The article "Gait Recognition for Lower Limb Exoskeletons Based on Interactive Information Fusion" was published in 2022. Journal: Appl Bionics Biomech.

# Gait Recognition for Lower Limb Exoskeletons Based on Interactive Information Fusion

**DOI:** 10.1155/2022/9933018

**Published:** 2022-03-26

**Authors:** Wei Chen, Jun Li, Shanying Zhu, Xiaodong Zhang, Yutao Men, Hang Wu

**Affiliations:** ^1^Tianjin Key Laboratory for Advanced Mechatronic System Design and Intelligent Control, School of Mechanical Engineering, Tianjin University of Technology, Tianjin 300384, China; ^2^National Demonstration Centre for Experimental Mechanical and Electrical Engineering Education, School of Mechanical Engineering, Tianjin University of Technology, Tianjin 300384, China; ^3^Institute of Medical Support Technology, Academy of System Engineering of Academy of Chinese PLA Military Science, Tianjin 300161, China

## Abstract

In recent decades, although the research on gait recognition of lower limb exoskeleton robot has been widely developed, there are still limitations in rehabilitation training and clinical practice. The emergence of interactive information fusion technology provides a new research idea for the solution of this problem, and it is also the development trend in the future. In order to better explore the issue, this paper summarizes gait recognition based on interactive information fusion of lower limb exoskeleton robots. This review introduces the current research status, methods, and directions for information acquisition, interaction, fusion, and gait recognition of exoskeleton robots. The content involves the research progress of information acquisition methods, sensor placements, target groups, lower limb sports biomechanics, interactive information fusion, and gait recognition model. Finally, the current challenges, possible solutions, and promising prospects are analysed and discussed, which provides a useful reference resource for the study of interactive information fusion and gait recognition of rehabilitation exoskeleton robots.

## 1. Introduction

In recent years, the number of patients with the motor function impairment caused by stroke, brain injuries, or Parkinson's disease steadily increased [1, 2]. Motor impairment has become the second leading cause of disability and death worldwide [3]. According to the WHO, stroke alone affects nearly half a million people a year in the United States and 11 million in Europe [4]. The majority of these patients have suffered from severe impairment of limb motor function, which affected their quality of life, preventing them from completing simple daily activities. The recent emergence of lower extremity rehabilitation exoskeleton robots has provided a track of hope for many patients with lower limb motor dysfunction, allowing them to practically return to normal lifestyles [5]. Rehabilitation programs targeting these patients which incorporate the patient gait personalization and movement intentions are the key to designing a proper lower extremity rehabilitation exoskeleton [6].

The article "Gait Recognition for Lower Limb Exoskeletons Based on Interactive Information Fusion" was published in 2022. Journal: Appl Bionics Biomech.

The application of gait recognition in the rehabilitation training of exoskeleton robot is rising in recent years. The initial research on gait recognition of lower limb exoskeleton only divided the simple gait stages through the original data or manually processed data [7–9]. Moreover, the gait information collected then is not sufficient and comprehensive enough to carry out effective gait recognition. The above research did not distinguish between patients with lower limb dyskinesia and healthy people, resulting in the slow progress of exoskeleton robot in rehabilitation training, while real-time gait recognition and adjustable motion posture will become the key link between these two different research groups. In order to recognize human motion patterns more comprehensively and reliably, it is necessary to consider the acquisition of human motion and interactive information, including various gait stages and complex physiological information [10].

With the rapid development of sensors and information technology, various information acquisition and fusion technologies are employed to complete more personalized gait recognition. These are mainly realized by means of limb motion information, plantar pressure and interaction force information, bioelectric information, and so on. The interactive information available for gait recognition is shown in Figure 1. Moreover, several machine learning methods appeared to replace the afore-mentioned techniques; some machine learning methods seem to replace the above technologies that mainly rely on manual feature extraction.

Currently, these commonly used adaptive pattern extraction methods mainly include support vector machine (SVM) [11], linear discriminant analysis (LDA) [12], Gaussian mixture model (GMM) [13, 14], artificial neural network (ANN) [15–17], hybrid algorithm [18], and other machine learning algorithms. For example, Zhang et al. integrated, analysed, and processed a variety of interactive information, which are then applied to study the gait recognition and associated algorithms [19, 20]. However, it is should be noted that majority of gait pattern recognition and classification algorithms are evaluated by the accuracy rate. Moreover, few people are involved in the generalization ability of the classifier model, which can reproduce the adaptability of machine learning algorithm to fresh samples. In the meantime, research related to the time efficiency of classification model, whether on training or test time, is even less.

The article "Gait Recognition for Lower Limb Exoskeletons Based on Interactive Information Fusion" was published in 2022. Journal: Appl Bionics Biomech.

With the deepening of the research on gait recognition of lower limbs, the manifestations of information have the characteristics of diversity, huge amount of information, and complexity of information relationship. Therefore, higher requirements are put forward for the timeliness, accuracy, and reliability of information processing [19]. As a new information processing technology, modal information fusion has gradually become a major progress in this field, providing a more accurate and personalized gait recognition pattern [21]. Information fusion is usually described as synthesizing information from multiple sources to obtain high-quality and applicable information. The schematic diagram of its standard gait recognition program is shown in Figure 2. For example, Chen et al. [22] combined plantar pressure and acceleration information, took advantage of SVM learning algorithm to identify five human motion gaits, and finally obtained a recognition accuracy of up to 94.08%.

The purpose of this paper is to provide a comprehensive review of the current status and development direction of the research on gait recognition of lower limb exoskeleton robots based on interactive information fusion in recent years. The main part of this paper, the overview of gait recognition, is divided into seven aspects: information acquisition, sensor placement on the human body, target group of information collection, biomechanics of lower limb exoskeleton, interaction in lower limb exoskeleton, interactive information fusion, and gait recognition model. Finally, the full text is summarized, and the corresponding solutions are proposed. This paper will provide a reference for the research of interactive information fusion and gait recognition of exoskeleton robot.

The rest of this paper is organized as follows: in Section 2, acquisition and analysis of interaction information is introduced. In Section 3, the research status of gait recognition in recent years is presented. Furthermore, in Section 4, the authors list the existing problems, including both technical and practical challenges. Finally, in Section 5, a conclusion of the full text is summarized.

## 2. Acquisition and Analysis of Interaction Information

As we all know, the research of lower limb exoskeleton robot is certainly inseparable from human participation. That is, when people wear exoskeleton robots to move, it is essential to collect, identify, and feedback human static and dynamic biological information [23]. Especially for the rehabilitation exoskeleton robot, it is obviously incomplete and unscientific to only consider the data of healthy people, because the user is a patient with limb dysfunction. Therefore, the rehabilitation training plan should fully consider the physiological factors of the patients, and even getting real-time gait information is the best choice.

The article "Gait Recognition for Lower Limb Exoskeletons Based on Interactive Information Fusion" was published in 2022. Journal: Appl Bionics Biomech.

### 2.1. Information Acquisition

In the research of exoskeleton robot, the common human biological information mainly consists of body movement information, plantar pressure information, interactive force information, and bioelectrical information. These signals can be regarded not only as the biological information of human body but also as the information transmission in the interaction between human body and exoskeleton robot. Because at this time, the human and the exoskeleton robot form a whole system, and these information and sensors act as perception system of the man-machine integration, which can sense the changes of the machine body and the external environment.

#### 2.1.1. Body Movement Information

The fast and effective acquisition of human body movement information is the first step of gait recognition research. Limb attitude information mainly comes from video image capture and inertial data acquisition.

Video-based motion capture system usually places reflective marks on the subject's skin or special clothing to capture human motion through camera and special software [24, 25]. The purpose of motion capture is to obtain the motion law of joints. There are three specific cases in the application of exoskeleton robot: (1) the need for bionic design [26]; (2) the generation and comparison of motion trajectories [27, 28]; and (3) the evaluation of real-time control and rehabilitation training [29, 30]. In the first case, the design parameters of an exoskeleton robot are provided by measuring human gait. In the second case, the motion data collected when the human body wears the exoskeleton robot are often compared with the control group without the exoskeleton robot [27]. Finally, in the third case, motion capture provides data for real-time control or evaluates the data of rehabilitation training.

However, it should be pointed out that the video-based gait capture equipment is expensive and complex to operate. In addition, the collected video image data is easy to be affected by factors such as illumination and activity range. Fortunately, wearable sensors such as gyroscopes, goniometers, and inertial measurement units can alternatively detect joint acceleration, velocity, and angular acceleration, so as to meet all the requirements of obtaining limb motion information. This method combined with other sensors is simple and easy to implement. Therefore, it has gradually become an important research direction of gait detection, recognition, and motion intention [31].

The article "Gait Recognition for Lower Limb Exoskeletons Based on Interactive Information Fusion" was published in 2022. Journal: Appl Bionics Biomech.

Moreover, the upcoming and popular commercial motion capture systems such as Xsens MVN [32, 33] and Xsens MTw Awinda have brought greater convenience to gait information acquisition, which not only overcome some of above limitations but also eliminate the errors caused by the external interference of the wearable sensors. It can be predicted that motion capture system will become the first choice for researchers to obtain gait information in the future because of its ease of use and analysis.

#### 2.1.2. Plantar Pressure Information

In the research of the perception of information acquisition of lower limb exoskeleton, the pressure-sensitive sensors are usually employed to determine and evaluate human locomotive gait and rehabilitation training [34]. Generally, the plantar pressure can be collected by force-sensing resistance sensors placed on the exoskeleton feet. According to the test needs, 2-5 or more sensors can be installed on the sole and heel of each foot to measure the pressure. Collecting plantar pressure information can distinguish swing and standing posture, identify walking gait [35], and monitor walking process [36]. By analysing the plantar pressure information, we can calculate the contact time between the foot and the ground and the time in the standing posture stage [37], identify the user's limb dynamic parameters [38], and judge the double standing posture, early swing, late swing, weight, and gait conversion [39]. In addition, plantar pressure can provide on/off signals to the controller or accurately compensate for the dynamic effects of torque measurement in swing motion [40].

#### 2.1.3. Interactive Force Information

After wearing an exoskeleton, the human body interacts with the exoskeleton. If plantar pressure refers to plantar pressure detection, the interaction force mainly emphasizes the relationship between force and reaction between human and exoskeleton. In order to obtain the interaction force between the body and the exoskeleton, Ma et al. [23] proposed to install a piezoelectric film sensor on the outer bandage of the lower limb rehabilitation robot. Similarly, Kyoungchul et al. [41] suggested placing the pressure-sensitive sensor on the thigh bracket; these sensors are employed to measure muscle movement and analyse the ratio between pressure and knee angle. In addition, De Rossi et al. [42] proposed a new interactive pressure measurement method based on soft silicon pressure sensor, which is located between the user and the exoskeleton robot. Compared with the most advanced measurement methods, the sensor is in direct contact with the wearer's skin, allowing distributed measurement of interaction pressure. Therefore, it can effectively improve the safety and comfort of human-computer interaction.

The article "Gait Recognition for Lower Limb Exoskeletons Based on Interactive Information Fusion" was published in 2022. Journal: Appl Bionics Biomech.

#### 2.1.4. Bioelectrical Information

The movement of human body is the result of the combined efforts of the brain, nerve, and muscle. The interaction of bioelectrical signals thus expresses the patient's needs and physical conditions. Electroencephalography (EEG) outputs are weak electrical signals generated by the electrical responses of brain nerve cell groups; the principle of the brain-computer interaction interface system is shown in Figure 3(a) [19]. However, due to the complexity, variability, and easy interference of brain computer interaction information, it is difficult to detect, save, and process it in real time, which limits its application in the gait recognition.

The surface electromyography (sEMG) signal is a superposition of motor unit action potential trains (MUAPT) generated during muscle contraction and can be obtained on the surface of muscles in a noninvasive way. Compared with EEG from the brain, sEMG signals are related directly to the limb's movements and have higher signal-noise ratio (SNR). That is to say, the sEMG signal can reflect not only the strength of muscle contraction but also the movement information of the joint. As a result, sEMG signals have been well applied in the recognition and prediction of human movement intentions, for instance, detection of sit-stand or stand-sit intentions [44] and prediction of the body's movement state, as well as the fatigue level and joint torque [45].  Figure 3(b) shows the acquisition method of sEMG interaction information. In addition, extracting sEMG signal as feedback command to study the motion control strategy of exoskeleton robot is also a research hotspot, which has been widely applied in rehabilitation exoskeleton robot [46].

In order to better identify the movement intentions of lower exoskeleton wearers, researchers have started to explore the neural interaction technology (i.e., neural stimulation). The basis behind the nerve stimulation is neuroplasticity, and its induction has an obvious beneficial effect on the rehabilitation [47]. Currently, the most common neural interaction technologies are biofeedback stimulation and electrical stimulation.

### 2.2. Sensor Placement on Human Body

In lower limb gait recognition, different parts of the body transmit different motion information, and this information has different effects on the recognition accuracy. Therefore, it is of great significance to find the gait information with the optimal recognition effect for human lower limb gait recognition. Sensor placement of all the studies covered in this review is presented in Figure 4. The purpose of this figure is to provide an overview of the distribution of lower limb sensor modules.

The article "Gait Recognition for Lower Limb Exoskeletons Based on Interactive Information Fusion" was published in 2022. Journal: Appl Bionics Biomech.

Kyeong et al. [57] found that an increase in the number of sensor locations and sensor types do not always lead to better results. Although the generated identification data set is more comprehensive and accurate, it significantly increases the data processing time and workload. Therefore, prior to the acquisition of perception information, it is necessary to evaluate the complexity of data processing and determine the optimal sensor position according to the results. In the above research, it is found that when observing the lower limb exoskeleton robot, the best sensor positions are mainly concentrated on the lower leg, thigh, and sole, while the sole sensors are mainly placed on the toes and heels.

Although as mentioned above, small changes in the direction and position of the sensor will affect the output of the sensor. In order to minimize the external disturbance to the gait information, the problem of sensor misplacement should be solved as much as possible. In addition to the initial calibration of the sensor before each experiment, researchers mainly take two methods to solve it. The first method is to find the best installation position of the sensor so that the sensor will not slide or move [62]. Secondly, the error caused by misplacement is compensated by an algorithm [63]. Some scholars also adopted an alignment method similar to borehole aiming to eliminate the influence of sensor misplacement, so as to solve the common misplacement problem of sensor [64].

### 2.3. Target Population of Information Collection

For lower extremity rehabilitation exoskeleton robots, most studies remain in the experimental stage. The users will most likely be patients with physical dysfunction, but a large proportion of the target population for gait recognition research are healthy adults, and it is obviously unreasonable to collect biological information only for healthy people [65, 66]. Ai et al. [10] took the physiological factors of the patients as the target population of experimental research to collect information and compare it with the normal walking of healthy people, which helps to improve the effect of gait recognition and rehabilitation.

Furthermore, in addition to healthy people and patients with lower limb dysfunction, the target population also includes people with weight-bearing. This is because whether it is power-assisted exoskeleton or rehabilitation exoskeleton, the wearer is equivalent to bearing the load brought by the robot's own weight and subject to certain constraints [10]. In the indoor environment, exoskeleton robots usually have corresponding devices to balance this load, but if they are outdoors or separated from the fixed device, the human body will still bear part of the weight. Therefore, it is of great significance to study the change of gait information after weight-bearing.  Table 1 shows the target population classification for information collection.

The article "Gait Recognition for Lower Limb Exoskeletons Based on Interactive Information Fusion" was published in 2022. Journal: Appl Bionics Biomech.

## 3. Gait Recognition Based on Information Fusion

The lower limb exoskeleton robot is a limb extension that fits closely with human. The physiological structure and biomechanical characteristics of human body should be fully considered in the design and test. Therefore, human biomechanics, human-computer interaction dynamics, and gait recognition models are the key problems that cannot be avoided in the research of rehabilitation exoskeleton robot. In the meanwhile, the gait and dynamics of exoskeleton robot are interrelated and interactive. Conversely, the accuracy of gait recognition is very important to improve the compatibility between the wearer and exoskeleton.

Furthermore, it is important to note that, although any of the sensor mentioned in Section 2 can measure human motion information, in order to obtain more accurate human motion gait, many scholars use the fusion technology of two or more sensors. With the development of sensor technology and information technology, collecting a variety of human information for fusion, analysis, and processing, and applying it to gait recognition, prediction, and real-time control of exoskeleton robot will be the development trend of rehabilitation exoskeleton robot.

### 3.1. The Lower Limb Exoskeleton Biomechanics

Walking is one of the main motions in the human-computer interaction of lower limb exoskeleton robot, which has a certain periodic motion law. Typically, a gait cycle is defined as the time between two heel landings. In a walking gait cycle, the lower limbs enter the support and swing stages alternately. The former accounts for about 60% of the gait cycle [73]. Each stage of the human gait cycle is shown in Figure 5.

Although a lot of achievements have been made in exoskeleton robot technology, the biomechanical mechanism of human wearing exoskeleton robot cannot be fully explained, and there is a lack of research on the interaction between human and machine. In recent years, the research on exoskeleton is no longer limited to the modelling of rigid components. Some scholars began to consider human factors and human-computer interaction and introduced human biomechanical models such as human muscle, bone, plantar, and their mutual constraints [74]. In fact, there are still many unknown areas to explore.

The article "Gait Recognition for Lower Limb Exoskeletons Based on Interactive Information Fusion" was published in 2022. Journal: Appl Bionics Biomech.

Nowadays, the biomechanical research related to exoskeleton robot mainly aims to achieve the following four purposes:

1. Bionic design [40, 75]: to get inspiration from the biomechanical research of human lower limb muscles, bones, and joints; to determine the degrees of freedom and the improvement of key parameter design and other details; and to complete the design of knee, ankle, hip, or leg. Some scholars even put forward the principle of structure matching and drive matching of lower limb exoskeleton robot [25]
2. Model accuracy [38]: to simplify the modelling of muscles and skeletal joints and to modify the rigid model of the original robot
3. Control design [76]: to add the biomechanical factors to the control algorithm
4. Performance evaluation [65]: generally, two or more groups of biomechanical data of human body are collected, one of which is the data after wearing the exoskeleton robot. The data of the latter group is employed to evaluate the correctness of the model or the working performance of the exoskeleton robot

The research target related to biomechanics mainly focus on the three groups of people: (1) healthy people [77]; (2) patients with lower extremity dysfunction [65, 66]; and (3) healthy people after weight-bearing [27, 78]. Among them, whether for an assist exoskeleton or a rehabilitated one, healthy people are often regarded as the benchmark or reference objects. In the second category, patients with brain injury and with spinal injury belong to this category. Analysing and evaluating the walking biomechanical behavior of these patients and comparing them with the normal walking of healthy people will help to modify the model and optimize the control of the rehabilitation robot. The third category is usually the research on the assist exoskeleton robots. No matter what kind of exoskeleton robot, in fact, this situation does exist.

In the above research, the research methods of biomechanics are as follows: (1) acquisition and analysis of various biomechanical parameters; and (2) establishment of human body local model. The human biomechanical parameters involved in the first method mainly include motion gait information, joint angle, joint driving force, joint torque, metabolic energy level, plantar pressure, sEMG signal, and other parameters [25, 65, 77, 79]. The second research method simplifies the modelling of muscles, bones, and joints. In fact, there is no mature method at present. For example, some studies have simplified the ankle joint as a variable stiffness actuator, and the knee joint and hip joint are designed as a series of elastic actuator [80].

### 3.2. Interaction in the Lower Limb Exoskeletons

As mentioned earlier, the exoskeleton robot is a tightly integrated human-machine system. It is often necessary to consider the interactive response of human body wearing exoskeleton to reflect the performance of exoskeleton robot. For the rehabilitation exoskeleton robot, the subjects of rehabilitation training are mostly paralyzed, stroke, and elderly patients. Not only the gait, movement, and plantar law are different from those of healthy people but also the biomechanics of muscle and bone and its biological response mechanism are completely different. Therefore, they cannot fully refer to the data of healthy people. Some research results have shown that the research on human-machine exoskeleton interaction is of great importance [79].

The article "Gait Recognition for Lower Limb Exoskeletons Based on Interactive Information Fusion" was published in 2022. Journal: Appl Bionics Biomech.

Currently, there is no plenty of research in this field. Some scholars have considered the local factors of human body and human-machine interaction and integrated them into the research of exoskeleton robot. Relevant research methods in healthy population include the following:

1. Establish a human-computer interaction model: using a spring-damping model or a combination of a nonlinear elastic and a viscoelastic element as a flexible connection at the contact point to express the interaction force [44]. This is followed by establishing the kinematic equation [37], and the referenced study has since been experimentally verified and evaluated [81]
2. Parameter comparison and adjustment: estimating the results and changes of internal force/torque based on the biomechanical models (for example, joints) and comparing them with experimental data [71]. Additionally, there are studies providing a way to identify the limb dynamics for each user, as well as parameters needed to accurately compensate for the dynamic torque measurement effects in oscillating motion [46].
3. Dynamic prediction and control compensation: based on the human-computer interaction model, a dynamic prediction and compensation motion control scheme is available [82]. Furthermore, several scholars have proposed a model for the interaction force estimation [83] and developed a system and program to estimate muscle fatigue through online physical interaction evaluation to provide mixed control of stimulated muscle performance [40]

For patients with lower limb dysfunction, achievements considering biomechanics and human-machine interaction are very rare. Research methods are generally limited to simulation or laboratory research, so as to try to adjust, modify, or optimize parameters or strategies on the results of human-machine interaction of healthy people, which is embodied in the following three aspects: (1) change parameters according to experimental tests [46]: force or driving torque, joint angle, and some studies can even optimize rehabilitation treatment schemes that can be customized for individuals [79, 84]; (2) design or add special components [75]; and (3) adjust the control strategy [76, 85, 86].

The article "Gait Recognition for Lower Limb Exoskeletons Based on Interactive Information Fusion" was published in 2022. Journal: Appl Bionics Biomech.

### 3.3. Interactive Information Fusion

As mentioned above, the exoskeleton robot perception system is an important subsystem for the wearer to perceive the external environment and transmit information. Therefore, it is very necessary for exoskeleton to obtain data by using various sensors, conduct rapid analysis and processing, and accurately recognize and control its movement. Currently, sensor fusion technology and deep learning are the research hotspots of exoskeleton robot, which will promote its development and is undoubtedly the trend of this field in the near future. The application of information fusion technology in gait recognition can be divided into three levels according to different levels of data abstraction.

#### 3.3.1. Data-level Fusion

Data-level fusion refers to the fusion on the original data layer, that is, the comprehensive information analysis performed by various sensors without a lot of preprocessing of the original information. Common applications include the combination of limb movement and plantar pressure interaction information, the fusion of plantar pressure and bioelectric information, or the fusion of the above types of information. As a matter of fact, an ideal exoskeleton perception and control system is to collect, fuse, analyse, and process all kinds of user information and apply it to the gait recognition, prediction, and real-time control of exoskeleton.

#### 3.3.2. Feature-level Fusion

Feature-level fusion refers to performing feature extraction by exploiting initial sensor information, allowing comprehensive feature information analysis and processing. As shown in Table 2, the feature extraction methods of feature-level fusion mainly focus on time-domain and frequency-domain analysis, which aims to quickly analyse and process data. For example, Zhang et al. [19] proposed that feature extraction has three main purposes as they studied gait recognition based on bioelectrical information: (1) reduce the dimension of sEMG signal; (2) reduce the complexity and classification of pattern recognition; and (3) improve efficiency. Luo et al. [20] calculated the root mean square and integral as signal features in sEMG gait phase recognition, in which the root mean square reflected the change of sEMG signal amplitude.

#### 3.3.3. Decision-level fusion

Decision-level fusion refers to extracting all kinds of feature information by making full use of feature fusion and adopting appropriate fusion technology according to the practical needs. Previous research on information classification and fusion system shows that data-level and feature-level information fusion can improve classification performance [93]. However, considering the large intraclass similarity and interclass variability among various signal classification types, for instance, Golrizkhatami and Acan [94] proposed an advanced fusion, which utilizes the majority voting mechanism to combine different classifiers to achieve decision-level fusion. The schematic diagram of the proposed method is shown in Figure 6. Generally speaking, compared with the other two fusion methods, decision-level fusion is a more complex and advanced fusion method.

The article "Gait Recognition for Lower Limb Exoskeletons Based on Interactive Information Fusion" was published in 2022. Journal: Appl Bionics Biomech.

For interactive information fusion, common fusion algorithms include Kalman filter [95], particle filter [96], complementary filter [97], and artificial neural network [98]. Generally, a single Kalman filter is not ideal, so the extended Kalman filter method or combined with other methods is a good choice [99]. In addition, from the perspective of sensors involved, a majority of research still choose wearable sensors to deal with gait information.

Table 3 lists the data fusion methods of multisensor at different levels in gait recognition. In fact, no matter what level of fusion method, there are limitations: (1) for data-level fusion: large amount of information processing and poor real-time performance; (2) for feature-level fusion: integration error and inherent sensor variance error make the deviation larger [100]; and (3) for decision-level fusion: the attitude phase detection characteristic of the sensor is an inherent characteristic that leads to the linear growth of integration error in attitude and position estimation [101].

The nice thing here is that more and more scholars started to try and even have adopted the deep learning method to fuse the information of exoskeleton robot in spited of the popular Kalman filter fusion method. Equally, with the development of deep learning, there will be a better way to process the video information. Consequently, in the face of the problem of wearable information acquisition or video acquisition, the deep learning method also puts forward a solution for the selection of sensors in the future. At that time, by means of deep neural network, the problem of image information fusion will be well solved.

Moreover, there is no unified data fusion theory and general fusion algorithm despite a large number of data fusion algorithms have emerged. Therefore, the current researchers concentrate their attention on developing simple and accurate algorithms to reduce the burden of calculation load and parameter adjustment [16].

The article "Gait Recognition for Lower Limb Exoskeletons Based on Interactive Information Fusion" was published in 2022. Journal: Appl Bionics Biomech.

### 3.4. Gait Recognition Model

#### 3.4.1. Feature Extraction

Before inputting the acquired gait information into the classification model, the most important step is feature selection. The quality of feature selection will directly affect the results of gait recognition. For nonwearable or wearable collection devices, the gait information is obtained in different ways, so the feature recognition methods are also different.

Firstly, for the gait information obtained from a nonwearable device, e.g., a video, model-based, and model-free gait feature extraction methods are available [112]. As mentioned above, the image features can be automatically extracted by convolutional neural network with the rise of deep learning technique [107, 108], which brings great convenience to feature extraction. Next, for the gait information acquired by wearable devices, there are many ways to apply to feature recognition, such as wavelet transform (WT) [113], principal component analysis (PCA) [114], fast Fourier transform (FFT) [115], and recursive feature elimination (RFE) [116]. These processes can be carried out in time domain [117], frequency domain, and time-frequency domain, respectively. The purpose is to select the optimal feature combination from the recognized features to improve the accuracy of gait recognition. Similarly, the deep learning network can also be employed to automatic feature extraction of signal processing [118], which is quite effective compared with the manual feature extraction of traditional machine learning algorithm.

#### 3.4.2. Recognition Methods

One of the most important features of lower extremity exoskeleton robot is the prospect of developing the intelligent human-machine cooperation. It can improve the rehabilitation effect by detecting the wearer movement intentions while requiring the robot control signal input to track the gait information and adjust in real time. Thus, accurate gait recognition is a crucial prerequisite. Due to impaired motor function, the patients' normal gait cannot be measured directly; therefore, it is necessary to carry out rehabilitation training and evaluate the normal gait data, which is of great significance in clinical application [119].

The gait recognition phases for lower exoskeleton robots are generally divided into five to eight stages. As shown in Figure 5, the typical five stages are the prestance, midstance, terminal stance, preswing, and terminal swing, respectively. In recent study, Yan et al. [120] divided the gait cycle into 4 stages and proposed a new voting weighting method to integrate the multidimensional acceleration signals collected by inertial measurement unit (IMU) into the voting-weighted integrated neural network (VWI-DNN) algorithm model and its classification accuracy, and Macro-F1 is up to 99.5%.

The article "Gait Recognition for Lower Limb Exoskeletons Based on Interactive Information Fusion" was published in 2022. Journal: Appl Bionics Biomech.

The gait recognition of lower limb exoskeleton generally includes normal walking, running, going up and down stairs, going up and down slopes, turning, and sitting-standing conversion. Semwal et al. [121] proposed a hybrid deep learning framework based on ensemble learning to recognize seven motion patterns: natural walk, standing, climbing stars, cycling, jogging, running, and knees bending, and the recognition accuracy reached 99.34%.

Numerous valuable computation methods of event and phase detection have been presented and adopted. These computation methods can be categorized into two main domains. One is the domain based on the threshold method, and the other is machine learning approach which is now among the most popular techniques to detect phases and events. The pie chat in Figure 7 illustrates the distribution of the detection algorithm in the reviewed papers. A large proportion of papers are on machine learning (73.9%), including traditional machine learning (26.1%), combined machine learning (13.0%), and deep learning (34.8%) in the pie chart.  Table 4 shows the application of some algorithms in phase recognition and behavior recognition. Although research results in gait recognition achieved by traditional machine learning algorithms such as support vector machine (SVM), Gaussian mixture model (GMM), and hidden Markov model (HMM) are not bad, the better and even optimized results have been continually obtained through the combined machine learning algorithms. In particular, the deep neural network has a surprising recognition effect on the gait information obtained by both wearable devices and visible cameras. Furthermore, the breakthrough technologies of real-time recognition algorithms have been embedded in the exoskeletons and achieved good effects, which undoubtedly promotes the favourable development of the lower limb exoskeleton robot.

It is worth noting that the sensor fusion method was also applied to study gait recognition in patients with hemiplegic stroke. The gait trajectory of the rehabilitation exoskeleton robot was calculated first, followed by the use of the zero movement point (ZMP) based on the semiactive control model trajectory [136]. The researcher's aim was to determine the patient movement intentions and deviations [84] to obtain an accurate gait recognition model based on the results.

#### 3.4.3. Interference Factors to Accuracy

It is worth emphasizing that in the above classification algorithm model, the recognition accuracy is difficult to reach 100%. The main reasons are as follows: (1) the gait information obtained by the classifier is not perfect, and the interference factors come from the gait information acquisition stage and information fusion stage. Wearable sensors are easily disturbed by misplacement [64], drift [137], noise [138], and other factors when acquiring gait information, resulting in the collected gait information is not pure enough. If these interference factors are not well preprocessed, such as filtering and denoising, it will lead to obvious integration error in information fusion. (2) Too few data sets are collected. In gait recognition, classifiers, especially neural network, need a large number of data sets for training to prevent over fitting. Therefore, researchers usually eliminate sensor integration errors through algorithms [139]. They continue to propose new classification algorithms [128] or integrate multiple classification algorithms [124] in order to continuously improve the recognition accuracy. (3) The classification algorithm still has defects. The traditional machine learning algorithm itself is not perfect, although it has achieved good recognition results in gait recognition. The development and application of deep learning techniques will be an effective way to solve this problem.

The article "Gait Recognition for Lower Limb Exoskeletons Based on Interactive Information Fusion" was published in 2022. Journal: Appl Bionics Biomech.

## 4. Challenges and Outlooks

In recent years, gait recognition of lower limb exoskeleton robot based on interactive information fusion has attracted extensive attention. Many scholars have carried out theoretical and experimental research in this field. However, the research on information acquisition, fusion, and gait of patients with lower limb dyskinesia is not mature and comprehensive, and there are still many problems and challenges. In the field of lower exoskeleton gait recognition, new interactive information detection technology is needed, mainly to improve the detection efficiency, so as to improve the wearer's comfort and rehabilitation effect. Similarly, the emerging advanced intelligent information fusion and gait recognition technology is also necessary, which can improve the compatibility between human body and exoskeleton. These new technologies and methods are expected to help the wearer or patients interact with the exoskeleton more effectively and also provide the basis for the design of follow-up control system and clinical rehabilitation training.

### 4.1. Information Acquisition Technology

The primary task of gait recognition of lower exoskeleton robot is to accurately and quickly detect and recognize the wearer's motion intention. In order to achieve this goal, several problems need to be considered: how to collect more accurate motion gait data and how to improve the comfort and usability of the wearer. Currently, in bioelectricity and wearable detection, EEG signal is weak and requires the wearer to pay high attention; sEMG and other similar limb information acquisition have some limitations such as lack of comfort and robustness, while video-based gait monitoring limits the range of activity.

The article "Gait Recognition for Lower Limb Exoskeletons Based on Interactive Information Fusion" was published in 2022. Journal: Appl Bionics Biomech.

To solve the above problems, a new high-resolution sEMG neural signal measurement system is developed to obtain accurate real-time human sEMG signals. This system is expected to achieve more accurate motion intention decoding through action potential extraction and motion unit decomposition [140]. Therefore, with the development of biological signal sensing technology, the prospect of implantable multichannel micronerve electrode array sensing technology will enable people to directly extract high-quality cortical electroencephalography (ECoG) from brain regions related to motor intention. In addition, it is believed that the design of interactive assistive technology in the future will more meet the needs, wishes, and abilities of wearers, and gait recognition and detection equipment also has the characteristics of simplicity, comfort, quietness, and acceptability [141].

### 4.2. Multimodal Information Fusion

According to the above analysis of this manuscript, the lower limb exoskeleton sensing system should have sufficient information acquisition, including not only human motion information and biological signals but also the interaction information between human and robot [119]. However, the more information collected is not always the better. It will increase the power consumption of the system and affect the efficiency of practical application [142]. Moreover, with the improvement and development of software and hardware algorithms such as data mining, signal fusion, machine learning, and deep learning, multimodal information fusion based on artificial intelligence is expected to become an important breakthrough in the future research direction of lower exoskeleton gait recognition, which is also an important means to realize human-computer interaction information fusion. It will be the research trend and goal of exoskeleton robot to comprehensively use multimode data for target classification and prediction, eliminate ambiguity and uncertainty, extract more effective data, and obtain more accurate motion gait recognition types through information complementarity.

### 4.3. Personalized Gait Recognition

With the development of exoskeleton technology, despite a lot of research on gait recognition, the results are still far from the emergence of mature products. In fact, gait analysis should fully consider the effects of physiological, psychological, pathological, and other factors of the wearer [24]. The existing data sets have a certain diversity in the walking environment, but it is still not flexible enough to reliably perform various gait analysis, and it is difficult to match the obtained gait patterns with personalized human motion. For example, the gait data provided in the current study are not sufficient to summarize the standard gait patterns of specific age groups, gender, or rehabilitated patients. In addition, the gait recognition method is only used for simple gait pattern recognition, such as standing, sitting, walking on the ground, and climbing stairs. According to literature reports, computer algorithm technology based on support vector machine and neural network has been widely used in gait analysis. To some extent, the ability of data analysis has been improved, but the system still cannot fully capture more personalized wearer gait patterns. As LeCun et al. [143] believe, the original form of processing natural data limits the traditional computing technology. Fortunately, deep learning can be employed to overcome the limitations of artificial engineering and will be more widely applied in gait data recognition, classification, and anomaly detection.

The article "Gait Recognition for Lower Limb Exoskeletons Based on Interactive Information Fusion" was published in 2022. Journal: Appl Bionics Biomech.

## 5. Conclusions

This paper summarizes the research status, progress, existing problems, and development trend of gait recognition of lower limb exoskeleton robot based on information fusion technology. Firstly, the common information acquisition methods, sensor placement, and target population of exoskeleton robot are discussed. Secondly, the research results of biomechanics and human-machine interaction that may be involved in the research of exoskeleton robot are reviewed and summarized. Furthermore, the specific applications, advantages, and disadvantages of data fusion, feature fusion, and decision fusion in gait recognition are described. In addition, the feature extraction and recognition methods of gait recognition model are commented. Finally, based on a large number of literature review, this paper also makes an extensive analysis and discussion on the limitations of sensor dislocation, lack of research on human-machine interaction, no uniform information fusion methods, recognition accuracy, and insufficient rehabilitation training and clinical practice. The challenges, application prospects, and solutions in information acquisition technology, multimodal information fusion, and personalized gait recognition are put forward. It is predicted that information fusion based on deep learning will be the research trend of exoskeleton robot gait recognition in the future. In conclusion, this review provides a useful reference resource for the research of interactive information fusion and gait recognition of rehabilitation exoskeleton robot.

The article "Gait Recognition for Lower Limb Exoskeletons Based on Interactive Information Fusion" was published in 2022. Journal: Appl Bionics Biomech.

## Figures and Tables

**Figure 1:** Tree diagram displaying available gait analyses.

**Figure 2:** Schematic diagram of a standard procedure implemented for gait recognition using data fusion. The acronyms used in this diagram correspond to the following: SVM: support vector machine; NB: Naive Bayes; LR: logistic regression; KNN: K-nearest neighbors; DT: decision tree; DA: discriminant analysis; GMM: Gaussian mixture model; ANN: artificial neural network; MLP: multilayer perceptron; PNN: probabilistic neural network; TDNN: time delay neural network; NLR: negative likelihood ratio; AUC: area under the curve.

**Figure 3:** Interactive bioelectricity information acquisition methods. (a) Brain machine interface system block diagram [43]. (b) Surface electromyography (sEMG) information acquisition [19].

**Figure 4:** Sensor positions [10, 17, 19, 48–61]. (a) Typical attachment positions of multiple sensors. (b) Type and location of the sensors applied in the papers (IMU: inertial measurement unit; FSR: force sensitive resistor; sEMG: surface electromyography, EEG: electroencephalography; MPJ: metatarsophalangeal joint).

**Figure 5:** Human gait movement cycle division [57].

**Figure 6:** The schematic of the method proposed in [88]. (ECG: electrocardiography.)

**Figure 7:** The distribution of detection algorithm in the reviewed papers.

**Table 1:** Classification of the target population for the information collection.

Target population	Sex	Age range	Average weight	Reference
Healthy people (6) Tibial amputee (3)	M (7) F (2)	21-34	61.25 kg	[67]
Healthy people (5)	M (3) F (2)	24-28	54.2 kg	[59]
Healthy people (4)	NA	21-27	73 kg	[57]
Healthy people (10)	M (10) F (0)	24-28	67 kg	[19]
Healthy people (4)	NA	20-27	NA	[17]
Healthy people (20)	NA	20-42	NA	[68]
Healthy people bearing loads (10)	M (10)	25-37	77.25 kg	[20]
Young people (41) Older people (41)	M (35) F (47)	24-76	NA	[69]
Older people (41)	M (16) F (25)	70-80	NA	[70]
Stroke patients (16)	M (12) F (4)	45-75	NA	[71]
Parkinson's patients (11)	M (8) F (3)	56-78	NA	[72]

**Table 2:** Feature-level extraction and fusion.

Original information	Method	Formula	Reference
sEMG Accelerometer	Root mean square (RMS)	$\text{RMS}=\sqrt{\frac{1}{N}\overset{N}{\underset{i=1}{\sum }}X_{i}^{2}}$	[20]
Accelerometer Angular velocity	Mean (*M*)	$M=\frac{1}{N}\overset{N}{\underset{i=1}{\sum }}X_{i}$	[87]
Accelerometer	Standard deviation (*σ*)	$\sigma =\sqrt{\frac{1}{N}\overset{N}{\underset{i=1}{\sum }}{\left(X_{i}-\mu \right)}^{2}}$	[88]
Accelerometer	Maximum (*X*_max_) Minimum (*X*_min_)	*X*_max_ *X*_min_	[89]
Accelerometer	Mean amplitude of peaks (*A*)	$A=\frac{1}{M}\overset{M}{\underset{i=1}{\sum }}X_{i}$	[90]
Accelerometer	Standard deviation magnitude (|*σ*|)	$\left|\sigma \right|=\sqrt{\sigma_{X}^{2}+\sigma_{Y}^{2}+\sigma_{Z}^{2}}$	[91]
Accelerometer Angular velocity	Correlation coefficients (*r*(*X*, *Y*))	$r\left(X,Y\right)=\frac{\text{Cov}\left(X,Y\right)}{\sqrt{D\left(X\right)D\left(Y\right)}}$	[92]

*N*: number of data samples; *i*:data sample index; *X*_*i*_: observation vector at *i*; *σ*_*X*_, *σ*_*Y*_, and *σ*_*Z*_ are the standard deviation values along the *x*-, *y*-, and *z*-axes, respectively.

The article "Gait Recognition for Lower Limb Exoskeletons Based on Interactive Information Fusion" was published in 2022. Journal: Appl Bionics Biomech.

**Table 3:** Fusion of multiple information sensors for exoskeletons.

Fusion method	Sensor type	Sampling rate	Fusion level	Real time/postprocessing	Purpose	Reference
NN	Encoder LBKA sensor sEMG	NA	Feature level	Real time	Ensure the success rate and reliability of intention detection	[102]
Filter selection Embedded selection	Vicon IMU	400 Hz	Feature level	Postprocessing	Effectively select a specified number of sensors	[103]
ZVU	IMU	100 Hz	Decision level	Real time	Determine the 3D attitude	[101]
Arbitration-based score-level fusion	Accelerometer	100 Hz	Decision level	Postprocessing	Improve recognition accuracy	[104]
EKF	Accelerometer Magnetometer Gyroscope	100 Hz	Data level	Real time	Solve sensor installation errors and path integral errors caused by sensor variance	[100]
RNN	ECG IMU	50 Hz	Feature level	Postprocessing	Improve robustness	[105]
NN	MMG sEMG	2048 Hz	Feature level	Real time	Joint torque prediction	[106]
CNN	Video	NA	Feature level	Postprocessing	Improve the effectiveness and robustness of gait recognition	[107, 108]
Markovian KF	Potentiometer IMU	50 Hz	Data level	Postprocessing	Reduce the IMU errors	[30]
Conjugate gradient algorithm	Accelerometer Gyroscope	100 Hz	Data level	Postprocessing	Find the minimum of the objective function	[109]
Multi-modality sensor fusion based on DL	FS AIS IMU	20 Hz	Feature level	Postprocessing	Overcome the challenge of gait classification from wearable sensors	[110]
LR	Accelerometer Gyroscope	40 Hz	Feature level	Postprocessing	Improve the detection and classification of STS	[111]

Note: The abbreviations in the table are reported in the Abbreviation section.

**Table 4:** Gait recognition methods of lower limb exoskeleton robots.

Recognition algorithm	Sensor type	Wearable/nonwearable	Real time/postprocessing	Gait recognition	Accuracy rate	Reference
SVMBP	FSR	Wearable	Postprocessing	Phase recognition	97.4593%	[122]
HMM	IMU	Wearable	Postprocessing	Phase recognition	91.88%	[123]
LDA KNN KSVM	sEMG EEG	Wearable	Postprocessing	Phase recognition	98.56 ± 1.34%	[124]
QDA	Accelerometer Gyroscope FSR	Wearable	Postprocessing	Phase recognition	>96.5%	[117]
DCNN	IMU	Wearable	Postprocessing	Phase recognition	97%	[125]
BLDA	Position sensor Interaction force GRF sEMG	Wearable	Postprocessing	Phase recognition	97.8%	[57]
ED-FNN	IMU FSR	Wearable	Postprocessing	Phase recognition	97.9 ± 0.1%	[126]
Ensemble learning-based hybrid deep leaning framework	IMU	Wearable	Postprocessing	Behavior recognition	99.34%	[121]
GMM	IMU	Wearable	Postprocessing	Behavior recognition	99.33%/ 95.75%	[127]
DDLMI	Accelerometer Gyroscope	Wearable	Real time	Behavior recognition	97.64%	[128]
SA-SVM	IMU FSR	Wearable	Real time	Behavior recognition	97.47±1.16%	[129]
IGPG	Motion capture system	Wearable	Real time	Behavior recognition	>97%	[130]
LMR	Onboard encoders Instrumented sensorized shoes	Wearable	Real time	Behavior recognition	99.4%	[131]
MvGGAN	Video	Nonwearable	Postprocessing	Behavior recognition	Higher accuracy	[132]
MCNN	Video	Nonwearable	Postprocessing	Behavior recognition	Higher accuracy	[133]
SCN	Video	Nonwearable	Postprocessing	Behavior recognition	89.8%	[134]
eMSM	Video	Nonwearable	Postprocessing	Behavior recognition	88%	[135]

Note: The abbreviations in the table are reported in the Abbreviation section.

The article "Gait Recognition for Lower Limb Exoskeletons Based on Interactive Information Fusion" was published in 2022. Journal: Appl Bionics Biomech.

## Abbreviations

NN: Neural network
LBKA: Length between the knee center of rotation and the ankle
sEMG: Surface electromyography
IMU: Inertial measurement unit
ZVU: Zero velocity updating
EKF: Extend Kalman filter
RNN: Recurrent neural network
ECG: Electrocardiography
MMG: Mechanomyography
CNN: Convolutional neural network
KF: Kalman filter
DL: Deep learning
FS: Floor sensor
AIS: Ambulatory inertial sensor
LR: Logistic regression
STS: Sit-to-stand and stand-to-sit transfers
SVMBP: Back propagation neural network based on support vector machine
FSR: Force sensitive resistor
HMM: Hidden Markov model
IMU: Inertial measurement unit
LDA: Linear discriminant analysis
KNN: K-nearest neighbor
KSVM: Kernel support vector machine
sEMG: Surface electromyography
EEG: Electroencephalography
QDA: Quadratic discriminant analysis
DCNN: Deep convolutional neural network
BLDA: Bayesian linear discriminant analysis
GRF: Ground reaction force
ED-FNN: Exponentially delayed fully connected neural network
GMM: Gaussian mixture model
DDLMI: Deep neural network-based deep location mode identification
SA-SVM: Simulated annealing algorithm-based support vector machine
IGPG: Individualized gait pattern generation
LMR: Locomotion mode recognition
MvGGAN: Multi-view gait generative adversarial network
MCNN: Multichannel convolutional neural network
SCN: Sequential convolutional network
eMSM: Enhanced mutual subspace method.
